RETRACTED

# The influence of the ultrasonic treatment of working fluids on electrospun amorphous solid dispersions

**DOI:** 10.3389/fmolb.2023.1184767

**Published:** 2023-05-10

**Authors:** Haibin Wang, Yingying Lu, Haisong Yang, Deng-Guang Yu, Xuhua Lu

**Affiliations:** ^1^ Department of Orthopaedics, Shanghai Changzheng Hospital, Naval Medical University, Shanghai, China; ^2^ Obstetrics and Gynecology Hospital, Fudan University, Shanghai, China; ^3^ School of Materials and Chemistry, University of Shanghai for Science and Technology, Shanghai, China

**Keywords:** blending electrospinning, nanocomposites, ultrasonic treatments, working fluids, amorphous solid dispersions

## Abstract

Based on a working fluid consisting of a poorly water-soluble drug and a pharmaceutical polymer in an organic solvent, electrospinning has been widely exploited to create a variety of amorphous solid dispersions However, there have been very few reports about how to prepare the working fluid in a reasonable manner. In this study, an investigation was conducted to determine the influences of ultrasonic fluid pretreatment on the quality of resultant ASDs fabricated from the working fluids. SEM results demonstrated that nanofiber-based amorphous solid dispersions from the treated fluids treated amorphous solid dispersions exhibited better quality than the traditional nanofibers from untreated fluids in the following aspects: 1) a straighter linear morphology; 2) a smooth surface; and 3) a more evener diameter distribution. The fabrication mechanism associated with the influences of ultrasonic treatments of working fluids on the resultant nanofibers’ quality is suggested. Although XRD and ATR–FTIR experiments clearly verified that the drug ketoprofen was homogeneously distributed all over the TASDs and the traditional nanofibers in an amorphous state regardless of the ultrasonic treatments, the *in vitro* dissolution tests clearly demonstrated that the TASDs had a better sustained drug release performance than the traditional nanofibers in terms of the initial release rate and the sustained release time periods.

## 1 Introduction

Modern science and technology have greatly promoted rapid developments in pharmaceutics for an “efficacious, safe and convenient” drug delivery, with pharmaceutical techniques and excipients as the focus (Feng, et al., 2022; Krysiak & Stachewicz, 2022; Wang et al., 2023a; Feng et al., 2023; Huang & Feng, 2023). New techniques, potential organic/inorganic excipients, and the related strategies are continuous reported (Chen, et al., 2022a; Zhu et al., 2022a; Meng, et al., 2022; Tang, et al., 2022; Wang & Feng, 2022; Wu, et al., 2022). Meanwhile, increasing efforts have been devoted to address enduring challenges, such as the dissolution and controlled release of poorly water-soluble drugs (Esim & Hascicek, 2021; Lv, et al., 2021; Murugesan and Raman, 2021; Sultana, et al., 2021). During the past few decades, many chemical methods (such as conjugation and chemical modification) and physical methods (such as melt extrusion, heat spraying, and encapsulation by beta-cyclodextrin, electrospraying) have been introduced into this application field (Wang, et al., 2019; Butreddy, et al., 2021; Al-Ghamdi, et al., 2022; Zhu, et al., 2022b; Shen, et al., 2022; Li, et al., 2023a; Lv et al., 2023a; Li et al., 2023b; Lv et al., 2023b). Among them, physical nano methods are gradually being applied in this field; bottom-up methods (such as molecular self-assembly) and top-down strategies (such as electrospinning and electrospraying) have frequently been investigated in recent years (Miar, et al., 2021; Chen, et al., 2022b; Shibata, et al., 2022; Xie, et al., 2022). For example, a simple search in Web of Science (2022–10–04) found 2,196 items when TS (topic) = “electrospinning or nanofibers” and TS = “poorly water-soluble drug or insoluble drug or solid dispersion” were exploited. Many reviews have been conducted on related topics (Wang, et al., 2021; Homaeigohar & Boccaccini, 2022; Pattnaik, et al., 2022; Raza Bukhari, et al., 2022; Wani, et al., 2022; Zhao, et al., 2022; Zhou, et al., 2022). The electrospun nanofibers loaded with a poorly water-soluble drug have different nomenclatures in different regions. In the region of electrohydrodynamic atomication, they are often called medicated nanofibers. In the field of polymer, they are frequently called as polymer-based nanocomposites. In textile field, they can be termed as non-woven mats. In pharmaceutics, they are essentially solid dispersions (SDs), in which the drug molecules are homogeneously dispersed all over the polymeric matrices (Chen, et al., 2022c; Liu, et al., 2023a).

RETRACTED

The knowledge and techniques about solid dispersions (SDs) are always being updated due to the continuous increase of poorly water-soluble drugs from high-throughput chemistry and bioengineering (Inocencio, et al., 2020; Bigogno, et al., 2021; Diogo and Ramos, 2022a; Diogo and Ramos, 2022b; Du et al., 2023a; Du et al., 2023b). In general, there are a series of factors that always co-act to ensure high-quality SDs for poorly water-soluble drugs. These factors include components and compatibility, morphology and structure, and physical forms of the loaded drugs (Paaver, et al., 2015; Ejeta, et al., 2022; Obeidat & Al-Natour, 2022). Particularly, natural source components, such as cellulose, chitosan, lignin, and polysaccharide, are the favorite polymeric carriers (Huang, et al., 2022a; Chen, et al., 2022c; Wang, et al., 2022; Liu, et al., 2023b). Pharmaceutical techniques are often a key element for ensuring acceptable SD compatibility between the drug and excipients, a favorable amorphous state (i.e., amorphous solid dispersions, ASDs), and reasonable morphology and structures for simple dosage transformations (Konda & Dhoppalapudi, 2022; Tan, et al., 2022).

Electrospinning (or electrostatic spinning), initially a textile method, is entering pharmaceutics, particularly the development of ASDs of poorly water-soluble drugs (in many publications, ASDs are called nano composites or molecular composites (Wang, et al., 2020; Kamali, et al., 2022; Liu, et al., 2022). This trend has a close relationship to the following capabilities of electrospinning: 1) Multiple components can be treated in a blended manner or a certain organized manner (such as core–sheath or side-by-side), provided that they can be co-dissolved into a certain solvent or solvent mixture (Zhang, et al., 2021; Zhu, et al., 2022c; Li, et al., 2022; Xu, et al., 2023a); 2) All kinds of nanostructures can be created in a single-step and in a forward straight manner, which holds great promises for productions on a large scale. These structures include monolithic, core–sheath, Janus, tri-layer core–sheath, tri-layer Janus, and combinations of core–sheath and Janus (Wang, et al., 2023b; Wang, et al., 2023c; Wang, et al., 2023d; Song, et al., 2023); 3) Extremely rapid transferring processes of the working fluids to solid nanofibers, which fall within the scope of a few tenths of a second. This means that the drug molecules are “frozen” in polymeric carriers in a homogeneous distribution state in the solid nanofibers, which is similar to the liquid working fluids (Huang, et al., 2022b; Brimo, et al., 2022; Wang, et al., 2023e). Thus, the electrospun drug-loaded nanofibers are molecular solid dispersions.

A common implementation procedure of the preparation of electrospun SDs is as follows: 1) a working fluid, mainly consisting of a functional ingredient (for applications of ASDs, this often means a poorly water-soluble drug) and a pharmaceutical polymer (sometimes also with a surfactant or other additives such as flavoring agents for oral administration) in an organic solvent (Han, et al., 2022); 2) electrospinning is implemented to prepare the medicated nanofibers; 3) medicated nanofibers are transferred into dosage forms for commercial products. In the first step, the key is that the drug and polymer must be co-dissolved in a certain organic solvent and must be compatible with each other; meanwhile, the polymer has fine electrospinnability and the loaded drug is appropriate for therapeutic treatments (Liang, et al., 2021; Ge, et al., 2023). For compatibility with biomedical applications, polymeric excipients from natural sources are more favorable (Abdalla, et al., 2020; Feng & Hao, 2021). There are many publications about case studies relevant to a certain drug or to a certain polymer, e.g., polyvinylpyrrolidone (PVP), which has been broadly explored as a drug carrier for enhancing the dissolutions of near 200 poorly water-soluble drugs in literature (Bikiaris, 2011; Chen, et al., 2022c). In the second step, although some efforts have been devoted to optimizing the electrospinning processes, many details are still often ignored, particularly by inexperienced researchers. These details include the preparation of working fluids, arrangements of the electrospinning apparatus, the collection of nanofibers, and the optimization of a series of working parameters, and even the safety issues associated with the implementations of an electrospinning procedure (Yu, et al., 2023a; Yu, et al., 2023b). Among them, some small details seem of little significance, but the real result is just the opposite, e.g., the ultrasonic treatments of working fluids before they are loaded into the syringes for electrospinning (Partheniadis, et al., 2022). However, very limited reports about how to prepare the working fluid in a reasonable manner are discussed in the literature. Thereby, an investigation was conducted to disclose the influences of ultrasonic pretreatment on the quality of resultant ASDs from the working fluids.

RETRACTED

In the present investigation, a working fluid composed of keteprofen (KET) as a model poorly water-soluble drug and ethyl cellulose as a drug carrier and the filament-forming polymeric matrix was prepared. Ethyl cellulose (EC) is a derivative of cellulose, which is a popular source for other drug carriers to modify controlled drug release profiles (Ahmadi, et al., 2022; Olechno et al., 2022; Yu & Zhao, 2022; Yao et al., 2023). The working fluid was divided into two sections: one was treated using ultrasonic waves before electrospinning, and the other was directly electrospun into nanofibers. They were compared in a series of characterizations to disclose the profound influences of the ultrasonic treatment on the quality of resultant nanofibers from several different standpoints.

## 2 Materials and methods

### 2.1 Materials

EC was obtained from Shanghai Haosheng Bioengineering Company (Shanghai, China). KET (white powders with a purity of 98%) was bought from Hengrui Pharmaceutical Company (Nanjing, China). The organic solvents of anhydrous ethanol and dichlorometahne (DCM) were purchased from Shanghai Merck Co., Ltd. (Shanghai, China). All other chemicals were of analytical grade, and water was double-distilled immediately before usage.

RETRACTED

### 2.2 Preparing fibers

A 6.0 g sample of KET was placed into a 100 mL solvent mixture of ethanol and DCM (v:v, 7:3) to form a drug solution. Subsequently, 22.0 g EC powder was placed into the drug solution. Mechanical stirring was performed for over 10 h to promote the dissolution of EC and homogenization of the co-dissolving solution. Two batches of the solutions were prepared in parallel. One of them was directly electrospun into nanofibers. The resultant nanofibers were termed as the traditional nanofibers F1 or amorphous solid dispersions (ASDs). The other nanofibers were treated using ultrasonic waves in an ice-water bath for 5 min, and later were subjected to electrospinning. The resultant nanofibers were termed as nanofibers F2 or treated amorphous solid dispersions (TASDs).

A BKE-1004DHT Digital Display Ultrasonic Cleaning Machine (with a power of 200 W and an ultrasonic frequency of 40 kHz, HangZhou Boke Ultrasonic Equipment Co., Ltd., Hangzhou, China) was exploited to conduct the ultrasonic treatment. The water bath had a size (lenght×width×hight) of 300 × 240 × 150 cm^3^. The samples were directly fixed in the bath with the water level higher than the level of electrospinnable fluids.

The working fluids were carefully loaded into a 10 mL syringe, which was fixed on a Cole-Parmer fluid driver. A blunt needle (G21) was utilized as the spinneret. The electrospun nanofibers were deposited on a collector, which was 20 cm away from the nozzle of spinneret and composed of an aluminum foil around a hard cardboard. After some pre-experiments, the applied voltage and the fluid flow rate were fixed at 14 kV and 2.0 mL/h, respectively. All the preparations were conducted at the ambient conditions (i.e., about a relatively humidity of 54% and a temperature of 22 °C.

### 2.3 Characterization

#### 2.3.1 Morphology

The prepared nanofibers were assessed using a scanning electron microscope (SEM, Quanter 450, FEI, United States). The samples were cut from the deposited nanofiber mats, and bound on a conductive adhesive to receive the sputtering of gold. The images were recorded under an applied voltage of 10 kV at different magnifications. The average diameters were estimated using ImageJ software (NIH, United States) by randomly selecting approximately 100 locations in the SEM images.

#### 2.3.2 Physical state

The amorphous state was measured using the X-ray diffraction (XRD) patterns. The raw powders of EC, KET, and their F1 and F2 nanofibers were measured in the 2θ range of 5°–60°. A Bruker X-ray diffractometer (Karlsruhu, Germany) with CuKα radiation was operated in the conditions of 40 kV and 30 mA.

RETRACTED

#### 2.3.3 Spectroscopical characterization

Attenuated total reflection–Fourier-transform infrared (ATR–FTIR) spectroscopy was utilized to determine the compatibility between EC and KET in the electrospun nanofibers. A Spectrum 100 FTIR Spectrometer (PerkinElmer, Billerica, United States) was employed at a range of 500–4,000 cm^-1^ with a resolution of 2 cm^-1^.

#### 2.3.4 Encapsulation efficiency

The KET entrapment efficiency (EE%) was measured using the following steps: the medicated nanofibers were accurately weighed and extracted in anhydrous ethanol. The solution was diluted using distilled water. The absorbance was measured at *λ*_max_ = 260 nm with a UV–vis spectrophotometer (UV-2102PC, Unico Instrument Co. Ltd., Shanghai, China). The KET contents in the nanofibers were calculated through the pre-determined calibration equation. Thus, the EE% can be determined with the following equation:

$$EE\left(\%\right)=\frac{W_{m}}{W_{c}}*100$$

where W_m_ represents the measured KET contents in the electrospun nanofibers and W_c_ is the originally added KET for preparing working fluid. All measurements were repeated three times.

#### 2.3.5 *In vitro* dissolution experiments

The KET release profiles from the medicated nanofibers were assessed in phosphate buffer saline (PBS). The basket method in the *Chinese Pharmacopoeia* (2020 Ed.) was adapted. Approximately 200 mg nanofibers was placed into 900 mL PBS, and kept at 37 °C and a rotation rate of 50 rpm. At predetermined time points, a 5.0 mL aliquot was withdrawn, and 5.0 mL of fresh PBS was added. The absorbance at *λ*_max_ = 260 nm was measured, and the amounts of KET could be calculated. All experiments were repeated six times.

#### 2.3.6 Statistical analysis

The results from the *in vitro* dissolution tests of F1 and F2 nanofibers were analyzed using one-way ANOVA. The threshold significance level was set at 0.05. Thus, *p* (probability) values lower than 0.05 were considered statistically significant.

## 3 Results and discussion

### 3.1 Improvements in the electrospinning processes from a standpoint of working fluid

The electrospinning process is only one step, and the nanofibers are generated in a straightforward and direct manner (Kang, et al., 2020; Sivan et al., 2022a; Xu et al., 2023b). The working fluids are transferred into solid nano products within several milliseconds. Many improvements have been reported in the literature about how to ensure the creation of high-quality nanofibers through a single step. These improvements mainly concern the electrospinning apparatus and the matching of different experimental parameters (Sivan, et al., 2022b; Jiang, et al., 2022); however, very limited attention has been paid to how to prepare a suitable working fluid, except for properties of electrospinnability and electrospinnable windows (Cao, et al., 2022; Huang, et al., 2022c; Lifka, et al., 2023). Meanwhile, when the properties of working fluids are discussed, their viscosity, surface tensions, conductivity, and rheological properties are frequently investigated. The influences of bubbles in working fluids seem be ignored. In this study, a co-dissolving fluid consisting of EC and KET was prepared. The KET was first dissolved into the solvent mixture of ethanol and DCM. Subsequently, EC was placed into the drug solution. Additionally, the blended solution was stirred for 24 h. Enough time was left to let the polymeric molecules absorb solvent, swell, disentangle, and dissolve into the solvents to obtain a homogeneous working fluid.

RETRACTED

Subsequently, the working fluids were divided into two sections, as shown in Figure 1. The application of ultrasonic treatment on the working fluid implemented an electrospinning process which created nanofibers with a higher quality and the corresponding improved sustained drug release performance. One section was treated with ultrasound (2 MHz) exposure for 5 min in an ice-water bath, and the other section was directly electrospun. The resultant nanofibers were denoted as F2 and F1 nanofibers, respectively. These two kinds of nanofibers were compared in terms of their morphologies, properties, and sustained drug release functional performance.

**FIGURE 1:** The application of ultrasonic treatment on the working fluid for implementing an electrospinning process to create nanofibers with a higher quality and the corresponding improved sustained drug release performance.

### 3.2 The influences on the morphologies of the electrospun nanofibers resulting from the ultrasonic pretreatment of the working fluids

Figure 2 shows SEM evaluations of the created nanofibers. The morphologies and diameter distributions of the F1 nanofibers that were fabricated from the working fluid without the ultrasonic pretreatment before electrospinning are exhibited in Figures 2a1–2a3. The assessment results of the F2 nanofibers produced from the treated working fluids using ultrasonic waves are exhibited in Figures 2b1–2b3. Under a larger magnification of ×80,000, the surface morphologies of F1 nanofibers (Figure 2a2) and F2 nanofibers (Figure 2b2) are more easily discerned than those in Figures 2a1–2b1.

**FIGURE 2:** The morphologies and diameter distributions of the nanofibers: **(a1–a3)** F1 nanofibers prepared from the working fluids without ultrasonic pretreatment; and **(b1–b3)** F2 nanofibers produced from the treated working fluids using ultrasonic waves.

RETRACTED

In comparison, they exhibit the following differences: 1) F2 nanofibers have a smoother surface than F1 nanofibers, which were bumpy and rough; 2) F1 nanofibers had a broader diameter distribution (830 ± 150 nm, Figure 2a3) and a slightly larger average diameter than F2 nanofibers (720 ± 110 nm, Figure 2b3); 3) F1 nanofibers had some nanofibers with a very small diameter. These differences are closely related to the profound influences of bubbles in the working fluids on the working processes.

Under ideal experimental conditions, the electrospinnable working fluids would be in a homogeneous state and should experience continuous and stable drawing by the electric forces, which result in homogeneous solid nanofibers with a uniform distribution of diameters. When the ultrasonic waves were explored to treat the working fluids, the embedded bubbles were repelled and the working fluids were close to continuous and homogeneous states. Thus, the resultant F2 nanofibers were smooth and straight, and had a uniform diameter distribution. However, when the working fluids were directly subjected to the electrospinning drawing, the embedded bubbles exerted profound impacts on the bending and whipping processes, which, in turn, impacted on the quality of the formed nanofibers.

Figure 3 is a diagram showing the influences of the embedded bubbles on the electrospinning processes. At different places of an ongoing unstable bending and whipping region, the embedded bubbles demonstrated their different influences. In the Taylor cone and straight-line steps, the influences of embedded bubbles should be very small due to the small volume and the relatively stable state of bubbles. At the early stage of the unstable bending and whipping drawings, the fluid jets still have enough solvent to maintain a “liquid” state to hold the bubbles. When the embedded bubbles are repelled to the ambient surrounding, these bubbles may result a sub-division of electrospinning, i.e., case “A” in Figure 3. These electrospinning sub-divisions should create nanofibers with a very smaller diameter, and greatly increase the diameter distribution of F1 nanofibers. This phenomenon can be deduced from the “bubble electrospinning” (Yang, et al., 2009; Li, et al., 2015) and “nano spider” (Wang, et al., 2011; Zhang, et al., 2020) processes reported in the literature.

**FIGURE 3:** The different influences of bubbles in the working fluids on the electrospinning processes and the related mechanisms that deteriorate the nanofibers’ quality: **(A)** resulting in new electrospinning; **(B)** making the fluids more winding; and **(C)** generating a crude surface morphology.

RETRACTED

In the middle of the unstable region, the surfaces of the fluid jets were turned to a semi-solid state. When the bubbles are repelled to the atmosphere, this may lead to the additional winding of fluids, and, in turn, result in more curved nanofibers. This is shown as case “B” of Figure 3. Throughout the unstable region, some of the tiny bubbles may have been retained in the fluid jets. In the final stage of the bending and whipping drawings and the subsequent deposition of solid nanofibers on the collector, these tiny bubbles may escape to the atmosphere, by which the collected nanofibers may collapse due to atmospheric pressure. This is one of the most important reasons why the F1 nanofibers exhibited a crude surface morphology with many bumps and holes, i.e., case “C” in Figure 3. In all of the above-mentioned influences, they are negative and would finally deteriorate the nanofibers’ quality.

### 3.3 The amorphous state of drugs presented in nanofibers from the same working fluids, with and without ultrasonic treatments

The amorphous status of poorly water-soluble drugs is favorable for their dissolution and diffusion to be release from their carriers. This is because they are in a highly energetic and disordered forms. When electrospun nanofibers are exploited as ASDs, on the one hand, they have their unique advantages and could expand their applications in many fields such as food, cosmetics, nutraceuticals, or pharmaceutics; on the other hand, the compatibility between the guest drug and the host polymer is very important for keeping the stability of the ASDs (Becelaere, et al., 2022; El-Shanshory, et al., 2022). Thus, XRD and ATR-FTIR were performed to determine the state of components and their compatibility within F1 and F2 nanofibers. The results are presented in Figures 4A,B, respectively.

**FIGURE 4:** Physical state measurements and the compatibility between the drug and polymeric carrier: **(A)** XRD patterns; **(B)** ATR-FTIR spectra; and **(C)** molecular formula of EC and KET.

The sharp peaks in the patterns of KET (Figure 4A) indicate that raw KET powders are crystalline materials, whereas raw EC powders and F1 and F2 nanofibers have no sharp peaks but humps. These phenomena suggest that EC is an amorphous carrier, and when KET was encapsulated into the nanofibers, it lost its original crystalline state but was converted to an amorphous state. Similarly, the sharp peaks in the FTIR spectra of KET almost disappeared in the spectra of F1 and F2 nanofibers in Figure 4B. A KET molecule has one -OH group and two -C=O groups. An EC molecule has many -OH groups. Thus, in the raw KET powders, the KET molecules are drawn together through hydrogen bonding to form crystalline particles. However, when KET molecules are distributed all over the EC matrix by the extremely fast drying process of electrospinning, KET molecules can be stably “hung” on the EC molecules by hydrogen bonding. Meanwhile, the steric hindrance of EC molecules and other secondary interactions such as hydrophobic and van der Waals interactions would impede the gathering of KET molecules. Thus, the KET molecules are distributed in the EC fibers in a molecular scattering state, i.e., an amorphous state. The ultrasonic treatments on the working fluids have no influence on the physical state of components in fibrous ASDs and their compatibility.

RETRACTED

### 3.4 Sustained release performance from the different amorphous SDs and the key mechanisms

The measured drug concentrations of KET in the solid F1 and F2 nanofibers were 21.71% ± 0.75% and 21.34% ± 0.86%, respectively. The theoretical calculation value according to the experimental conditions was 21.43%. Thus, the encapsulation efficiency (EE, %) of F1 and F2 nanofibers were 101.31% and 99.58%, respectively. Just as anticipated, the ultrasonic treatments on the working fluid resulted in no drug loss.

The homogeneous distribution of KET molecules within the EC matrices can benefit a stable and continuous release, which is a key application of ASDs as sustained drug release materials. The *in vitro* drug release characterizations of F1 and F2 nanofibers are presented in Figure 5A. Both nanofibers could exhibit typical sustained drug release behaviors. The statistical analysis results indicated that *in vitro* dissolution profiles of F1 and F2 nanofibers were significantly different. In another expression method, an interpolation technique was exploited to achieve the time points that were needed for releasing a certain percentage of the loaded drug. The results are included in Figure 5B. Clearly, the F2 nanofibers, i.e., the TASDs, demonstrated better sustained drug release performance than the F1 nanofibers, i.e., the ASDs. This judgement can be reached from two aspects: one is the longer sustained release time periods for release percentages of 50% and 90% (2.87 vs 1.72 h and 14.61 h vs 10.18 h, respectively); the other reason is a smaller initial burst release. A 30% release in 1 hour is commonly regarded as a standard line for judging initial burst release. The F1 nanofibers took only 0.49 h to release 30% of the loaded KET, suggesting a more severe initial burst release than F2 nanofibers.

**FIGURE 5:** The sustained release performance of the F1 and F2 ASDs: **(A)** *in vitro* dissolution tests; **(B)** the time needed for releasing a certain percentage of the loaded drug; and **(C)** the drug release mechanisms regressed according to the Peppas equation.

RETRACTED

The Peppas equation (Peppas, 1985) is exploited to evaluate the drug release mechanisms from the two kinds of nanofibers. The regressed equations are included in Figure 5C. For F1 and F2 nanofibers, their results are listed as the following Equation 1 and (2), respectively.

$$L\text{og}\left(Q_{1}\right)=1.61+0.34\mathrm{Log}\left(t\right)\;\left(R=0.9965\right)$$ (1)

$$L\text{og}\left(Q_{2}\right)=1.51+0.38\mathrm{Log}\left(t\right)\;\left(R=0.9969\right)$$ (2)

These results indicate that KET was releases through a typical Fickian diffusion mechanism from both F1 and F2 nanofibers, as suggested by the power exponent values of 0.34 and 0.38, smaller than the judgement value of 0.45. Thus, the ultrasonic treatment had no influence on the drug release mechanisms from the final electrospun products.

Thus, the key is that there are several factors of nanofibers’ morphologies, which can exert their influences on the release behaviors of drug molecules (diagrammed in Figure 6). These factors include nanofibers’ diameters and size distributions (Figure 6A), breaking possibility (Figure 6B), and smoothness of surface (Figure 6C). Compared with F1 nanofibers, F2 nanofibers had a more uniform diameter distribution, a smaller breaking possibility, and a smoother surface. These factors acted together to ensure them a better drug sustained release profile. Particularly, the F1 nanofibers had a surface full of bumps and hollows, which not only increased the surface area, but also shortened the diffusion route of drug molecules, which was extremely unfavorable for an extended release. Today, multiple-functional nanomaterials are desired in many fields, particularly in biomedical applications (Li, et al., 2023c; Wang, et al., 2023f; Qi, et al., 2023; Zhang, et al., 2023). The combination of a deep understanding of the materials conversion processes and a clear knowledge about the molecular mechanism of biomedical action is able to promote the developments of many novel biomedical products with an obvious process-property-performance relationship.

**FIGURE 6:** The influences of ASDs’ morphologies on the drug release behaviors: **(A)** the increased surface area; **(B)** possible breaking of nanofibers in the curved places; and **(C)** increased surface area from the uneven surface and shortened diffusion distance of the drug molecules.

## 4 Conclusion

With EC and KET as the drug carrier and active ingredient, respectively, two kinds of amorphous solid dispersions were prepared from the same working fluids using electrospinning. Before electrospinning, one of the working fluids was treated using ultrasonic waves for 5 min and later converted into F2 nanofibers; the other was directly electrospun into the traditional nanofibers F1. XRD and ATR–FTIR clearly demonstrated that both F1 and F2 nanofibers were amorphous solid dispersions and the drug and carrier had good compatibility. However, SEM results revealed that the F2 nanofibers from the fluids treated with ultrasonic waves were of better quality than those from the untreated fluids in terms of linear morphology, smooth surface, and diameter distribution. Furthermore, the *in vitro* dissolution tests verified that the F2 nanofibers could provide a better sustained drug release performance than nanofibers with a smaller initial burst release and a longer sustained release effect.

RETRACTED

In this study, one of the most common poorly water-soluble drugs, KET, and one of the most common polymeric excipients, EC, were selected as a model drug and a filament-forming polymeric matrix, respectively, to determine the profound influence of embedded bubbles in working fluids on the electrospinning processes, the resultant nanofibers, and their controlled drug release performance. ASDs are always a focus for resolving the dissolution of poorly water-soluble drug. The disclosed strategy based on these common materials should make it suitable and useful to develop many other sorts of novel ASDs for promoting the dissolution of poorly water-soluble drugs or modifying their release profiles. Meanwhile, the protocols reported here should be a good reference for how to optimize the experimental procedures for creating high-quality nanofibers, and how to evaluate potential nanofiber-based products in future.

## Data Availability

The original contributions presented in the study are included in the article/Supplementary Material, further inquiries can be directed to the corresponding authors.
